The article "Regulation of Tumorigenesis in Hepatocellular Carcinoma via the AKT3 Pathway in Cell Lines" was retracted in 2023. Reasons: signs of a paper mill; compromised peer review; unreliable results or conclusions.

# Regulation of Tumorigenesis in Hepatocellular Carcinoma via the AKT3 Pathway in Cell Lines

**DOI:** 10.1155/2021/3267536

**Published:** 2021-10-28

**Authors:** Mingxuan Xing, Xinwei Xie, Zhi Liu, Xiaohong Du

**Affiliations:** Department of Hepatobiliary and Pancreatic Surgery, The First Hospital of Jilin University, Changchun, 130021 Jilin Province, China

## Abstract

**Background:**

The estimation of hepatocellular carcinoma (HCC) is tremendously inferior because of the formation of chemoresistance, integrated with essentially increased stemness belongings. At present, the relevance between miR-122 and cancer development was mostly undisclosed with single study reflecting its importance in glioblastoma. *Material and Methods*. The research here was focused to investigate the task of miR-122 to modulate tumorigenesis in hepatocellular carcinoma by aiming AKT3 in the management of hepatocellular carcinoma stemness and chemosensitivity. The method of QRT-PCR was performed to investigate the aspect of miR-122 and AKT3 in tissue sample and cell lines. The evaluation was done using gain- or loss-of-function in order to retrieve the function of miR-122 in the hepatocellular carcinoma cells, including cell multiplication and stemness effects. The properties of hepatocellular carcinoma were discovered by the development of sphere development, cell feasibility, and the emergence of colony. RNA immunoprecipitation (RIP), luciferase reporter, and the RNA pull down evaluation were conducted to investigate the communication between the miR-122 and AKT3. Therefore, a naked mouse xenograft specimen was set up for the in vivo analysis.

**Results:**

Here, we determined the new role of AKT3 and unmediated target of miR-122. The reimposition of miR-122 appearance in the hepatocellular carcinoma cell lines reduces the levels of AKT3 and also hinders the relocation and expansion of cells by prompting apoptosis. These phenotypes are antitumor in nature and can be retrieved by the reorganization of the AKT3 expression which signals the crucial role of AKT3 in the miR-122 arbitrated HCC modification. The in vivo analysis demonstrated the reimposition of miR-122 entirely obstructing the xenograft expansion to manage tumorigenesis in hepatocellular carcinoma and a prospective remedial entrant for the liver cancer.

**Conclusion:**

In this study, it was observed that miR-122 encourages the stemness role of hepatocellular carcinoma and diminishes the chemosensitivity by cleaning the miR-122 in order to initiate the AKT3. The in vivo study reflected the restoration of miR-122 which completely hinders the xenograft growth to regulate the tumorigenesis in the HCC.

## 1. Introduction

One of the most frequently occurring liver malignancies is hepatocellular carcinoma (HCC) which is observed in approximately 75-85% of the cases. It is graded at the fourth position among the cancer cases and death related to them at global level [1]. The hepatocellular carcinoma usually appears from a long-term inflammatory medium which occurs because of various causes. MicroRNAs (miRNAs) are the little noncoded RNAs which behave as the medium of the RNA intrusion pathway to manage the protein expression by unsettling the hindrance of the target agent RNAs [2, 3]. Since the miRNAs generally hold their targets with insufficient complementarity, an individual miRNA might have numerous gene targets and multiple effectors in the same effective pathway, yielding a consistent physiological reaction through numerous equivalent uneasiness [4, 5].

Hepatocellular carcinoma (HCC) is ranked 5th in the usual cases of malignant tumor amongst men and 7th among the women at a global scale, which causes more than 700,000 mortality cases every year [6, 7]. Moreover, breakdown of hepatocellular carcinoma can be induced by collapse of untimely diagnosis, absence of the effectual therapeutic targets, and deficient observation. Thus, the formation of new diagnostic procedures and the recognition of the fresh targets for the remedial involvement are immediately required for the discovery and medication of the hepatocellular carcinoma [8, 9]. The persistent liver inflammation frequently causes the fibrosis proceeded by cirrhosis and eventually hepatocellular carcinoma. The modifications in the condition of the liver all over the formation of hepatocellular carcinoma are supported by altering the tumor microenvironment (TME) form that continues an opportunity advocating malignancy. The modification of the signaling pathways is general in hepatocellular carcinoma and is important for the development of the malignancy [10].

The protein kinase B (AKT/PKB) includes AKT1, AKT2, and AKT3 which are the prime interventions of signaling pathways which supervise the cellular procedure managing the cell size, growth rate, expansion, existence, glucose metabolism, and steadiness of genome. AKT3 is indicated in the brain and the testes. AKT comprises of three domains on constructional level: (1) PH domain of amino-terminal, (2) middle section distributing homology with other cAMP-dependent protein kinases, and (3) a carboxyl-terminal section performing as a controller domain [11]. These isoforms share homologies in their catalytic areas, but they separate in the PH and the control areas [12].

## 2. Material and Methods

Cell culture lines were procured from Thermo Fisher Scientific and very well preserved in DMEM (Dulbecco's modified Eagle's medium) with 10% FBS added with L-glutamine at 37°C with 5% CO_2_.

### 2.1. RT-PCR

Quantification of miR-122 expression levels was done for AKT1, AKT2, and AKT3 by RT-PCR TaqMan miRNA assays (Invitrogen). Complete RNA extraction was performed by Total RNA Isolation Kit MagMAX™ mirVana™ (Thermo Fisher) where it was reverse transcribed via the reaction mixture having miR-specific stem-loop RT primers.

Triplicate reactions were performed for qPCR (quantitative real-time polymerase chain reaction) with TaqMan and cDNA primers from the Universal Master Mix without adding AmpErase™ uracil N-glycosylase (UNG) (Fisher Scientific). At 950°C, qPCR was performed for a 10-minute duration which includes maintenance of 950°C temperature for 40 cycles for a duration of 15 seconds, 60 seconds cycle at 600°C in a 7900HT Fast Real-Time PCR System (Thermo Fisher Scientific) with cycles of threshold ABI PRISM® 7000 Sequence Detection System (Thermo Fisher).

Normalization of mRNA quantification data was done till 18S RNA. Expression of miRNA data was done in relation to RNU48 small nuclear (sn) RNA TaqMan PCR which was done on the same samples. The fold expression was done with 22DDCt method for mean CT values.

### 2.2. Animal Studies

Mice who were aged six to eight weeks were obtained for research purposes from Laboratory Animal Center of the Chinese Academy. Mice were kept in ventilated cages in animal facility. All procedures were approved by animal ethical committee as per Institutional Animal Ethical Guidelines. Establishing tumors in mice was done by injecting 5 × 10^6^ cells in 1 : 1 ratio by reconstituted basement membrane (Matrigel). The dimensions of tumors were measured via vernier calipers, and growth percentage was calculated. One-way ANOVA was used for statistical analysis where *p* < 0.001 is denoted by ∗∗∗.

### 2.3. Immunoblotting

Lysis of cells in a buffer was done which contained 50 mM NaCl, 50 mM HEPES, 1% Triton X-100, 1 mM PMSF, 1 mM b-glycerophosphate, 10% glycerol, 1.5 mM MgCl_2_, 0.5% NP-40, and 1 mM EGTA. Adding cocktail of protease and phosphate inhibitor (Cell Signaling Technology) was done prior to the use. Then, protein concentrations were determined in the protein assay as per instructions of the manufacturer. 30-50 mg protein was used via SDS-PAGE and then transferred into nitrocellulose membrane. Primary antibodies were used for detection of blots, posting that secondary antibodies were used for luminescence.

The proliferation, migration, and apoptosis of cell were performed via resazurin fluorescent assay. Cells were seeded overnight postincubation at 37°C in 5% CO_2_ where 3000–5000 cells/100 *μ*l/well were kept in DMEM with 10% FBS in a 96-well plate.

Fluorescent dye resazurin was added in a ratio of 1 : 1000 in each well. Incubation of cells was done for 4 hours at 370°C in 5% CO_2_ where fluorescence was induced. ELISA kits were also used for apoptosis. Coating of phosphorylated BAD (Abnova) and cleaved caspase 3 (Thermo Fisher Scientific) was done on microwells via the manufacturer. Coated antibodies were done via targeted proteins after incubation with the cell lysate. Then, a detection antibody was added for capturing the targeted protein. Recognition of bounded detection antibody was via HRP-linked secondary antibody. Then, cell migration assay kit was used in 24-well plate for polycarbonate membrane inserts. The cells which are migratory in nature are able to move towards hepatic growth factor via membrane pores, whereas the nonmigratory cells are extracted from the top surface of the membrane where these migratory cells are quantified and stained.

### 2.4. Evaluation with Luciferase Assay

Three days after the procedure of transfection with suitable establishment, the cells were made undergone and handled for luciferase luminescence quantification. The homogenous reagent system of Dual-Glo luciferase assessment (Promega) was utilized for identifying the luciferase action as explained by the maker. A suitable size of Dual-Glo substance was put into the cell element permitting the cell lysis and following discovery of firefly luminescence. The normalization of the specimens was executed by inclusion of the Dual-Glo Stop and Glo element which allowed the revelation of Renilla luminescence along with the luciferase action in the relative light units (RLU) which was thereafter computed.

### 2.5. Statistical Analysis

The quantification of the data was done via the mean ± SD. Student's *t*-test was used for determination of the difference between two groups significantly. Bonferroni was used as a post hoc test after one-way ANOVA, and significant differences were analyzed in various groups. *p* < 0.05 was considered as statistically significant.

## 3. Results

### 3.1. Binding of miR-122 to 3′-UTR of hsa-AKT3

The luciferase activity was also measured using Huh-7 and SNU-182 parenterally; the overexpression of GFP and miR-122-GFP caused transfection with vector alone or luciferase reporter 3′-UTR. The results were represented at various independent levels where the statistical significance was ^∗∗^*p* < 0.01 and ^∗∗∗^*p* < 0.005 (Figure 1).

### 3.2. Expression of AKT3 in miR-122 Levels for HCC Cell Lines

The expression of AKT3 is conversely related to levels of miR-122 in HCC cell lines of chronic hepatitis B virus. Expression levels of AKT3 and miR-122 were examined in human HCC cell lines and normal human liver. When the miR-122 expressions were estimated in HCC cell lines in comparison to normal liver, the levels were downgraded (Figures 2, 3, and 4).

The AKT3 expression levels are increased in SNU-182, Hep3B2, and SNU-475 with merely no or little miR-122 expressions (Figure 2). In the case of HCV-transformed Huh-7 line and HepG2 cell hepatoblastoma, there is no overexpression of AKT3 in the tissues when compared against normal liver tissues. Levels of Huh-7 AKT3 are not significant when miR-122 levels are considered endogenously. Due to the lack of binding site for miR-122, there is a slight increase in mRNA levels of AKT1 and AKT2 for cell lines when compared with a normal liver.

Similar results were noted in AKT3 transcript levels; protein levels of AKT3 were significantly larger than SNU-475 and SNU-182 HCC cell lines (Figure 5). All these results show that the levels of miR-122 level are inversely opposite to protein levels of AKT3 mRNA in HCC cell lines.

In in vitro cell proliferation, the overexpression of miR-122 inhibited the cell proliferation when the tumor growth was studied in a HCC SNU-182 xenograft model. The cell proliferation was measured for SNU-182, GFP, and miR-122 (Figure 6).

Cell migration inhibition in HCC lines where miR-122 expression was restored and induction of apoptosis happened. Antitumor activities were induced by AKT3 expressions (Figure 7). The measurement of phosphorylation of cleaved caspase 3, BAD, and total BAD in cells is shown in Figure 8.

## 4. Discussion

### 4.1. miR-122 Promptly Binds to the 3′-UTR of hs-AKT3 to Control Its Appearance

Initially, we validated that miR-122 is solely expressed in a standard human liver tissue by differentiating its appearance in other common tissues. Low expression of miR-122 in tumor cell lines from other organs, additionally assuring that miR-122 is a liver-specified miRNA as it is studied. The utilization of RT-PCR was also validated for miR-122 expression which was remarkably either downmodulated or entirely terminated in a range of human HCC lines comprising of SNU-182, SNU-475, and Hep-3B2 and also a hepatoblastoma cell line (Hep-G2). However, the expression of miR-122 sustained a remarkable level of miR-122 expression. Thus, the expression of miR-122 is particular to the liver and is extremely subdued in the human HCC cell lines.

As studied the regulatory behavior of AKT in various cancers, we determined to assess the course alignment between the AKT3 3′-UTR; it was observed that in three types, the human miR-122 reflects limited complementarity. Further, we expanded the human AKT3 3′-UTR by the PCR method and subcloned it as a luciferase reporter vector. This establishment was utilized for the cotransfection with the miR-122 establishment in SNU-182 and Huh-7 cell lines. Further, it was discovered by the luciferase assay whether miR-122 can combine to the 3′-UTR of AKT3. The outcomes indicate the diminished firefly luciferase action in the SNU-182 cells by the miR-122 expression which signals the binding of miR-122 to 3′-UTR.

### 4.2. The Downregulation of AKT3 by the Overexpression of miR-122 in HCC

Now, we inspected the consequences of miR-122 over appearance in the human HCC cell lines, Huh-7, SNU-475, Hep3B2, and SNU-182. The subcloning of miR-122 was done in a lentiviral appearance vector and was fortunately overexpressed in these cell lines. The overexpression of miR-122 diminished mRNA and the AKT3 protein levels in the SNU-182 cells. The equivalent data was assembled from the Hep3B2 and SNU-475. Some growth of miR-122 in Huh-7 cells was observed, and the expression of miR-122 diminished AKT3 levels which was noticed only on the immunoblot with lengthy duration of revelation because of the small endogenous levels of AKT3 in the cell line. We analyzed the modifications in the other AKT class members for validation in the miR-122-transduced cells. The AKT1 or AKT2 expression was not remarkably modified by the overexpression of miR-0122 in SNU-182 and Huh-7, thus indicating the precise targeting of miR-122 on AKT3. Consequently, the outcomes favor the theory of negative control of miR-122 on AKT3 conversion in the HCC cell lines.

### 4.3. The Hinderance of Cell Migration and Prompting of Apoptosis by Overexpression of miR-122

AKT kinase controls a variety of cellular approaches involving cell proliferation, presence, size and response to nutrient accessibility as well as angiogenesis and tissue capture of tumour cells. Consequently, we determined if the obstruction of AKT3 by reinstitution of miR-122 expression will result to antitumor effects in the SNU-475 and SNU-182 in contrast with the HCC cell line with the endogenous miR-122 expression. The Huh-7, SNU-182, and SNU-475 cells relocate across the polycarbonate membrane on stimulation of HGF-1, a well-formed characteristic of extremely modified HCC cells. The HGF-induced cell relocation in the HBV-altered SNU-182 and SNU-475 is reduced by the overexpression of miR-122, which signifies the relocation in SUN-182 and SUN-475.

The overexpression of miRNA-122 does not change the cell migration in the Huh7 cells. We conducted an experiment to confirm that the miR-122 convinced hinderance in the cell relocation occurs because of the reduced level of AKT3 in the SNU-475 and SNU-182 cells. In this experiment, we temporarily transfected a vector, thus encoding the human-based AKT3 cDNA in the SNU-182, that secured the GFP or miR-122-GFP. The outcomes signify the unstable overexpression of the AKT3 in the miR-122-GFP expressing the SNU-182 cells liberating the relocating hinderance reporting the above by 70% (approx.). The migration assays indicate that miR-122 overexpression in the SNU-182 cells reduces the AKT3, causing the obstruction of HGF-induced resettling of cell in SNU-182 cells. Moreover, the obstructed miR-122 migratory reactions were saved by unbalanced restoration of the AKT3 expression. Consequently, miR-122 control of the AKT3 expression is obligatory and adequate in balancing the HCC cellular relocation in the HBV-altered cells.

### 4.4. The In Vitro and In Vivo Antitumor Actions Are Prompted by the Overexpression of miR-122 in the Energetic HCC Cell Lines in the SNU-182 Cells

Here, we investigate the outcomes of miR-122 on the cell multiplication after assessing the regulation of the apoptotic pathways by the miR-122 in the HCC cell lines. As per the estimation from our apoptotic assays, the overexpression of miR-122 reasonably paced down the growth of cells in the SNU-182 but not in the Huh-7. The obstruction of cell growth was saved by the abnormal expression of AKT3 in the miR-122 fostering the SNU-182 cells.

The deficiency of control actions was identified in Huh-7 cells with the overexpression of miR-122, which may again be conducive to regulate the endogenous miR-122 expression in these cells signifying that growing miR-122 expression in these cells is not enough to modify the tumorigenic characteristics. Eventually, we analyzed the outcomes of miR-122 overexpression upon the in vivo expansion. The SNU-182 cells securely overexpressed miR-122-GFP were formed and inserted in a nude mouse, thus observing the progress of the tumor over the period of time.

A substantial downregulation of miR-122 has been previously demonstrated in many HCCs and usually reflects the below standard prognosis, thus indicating the higher risk of metastasis. This research inspects the role of miR-122 in the process of tumorigenesis of the HCCs. Here, we even exhibit the tumor suppressor role of miR-122 in the HBV-altered HCC cell lines and broadcast AKT3 as the new and unmediated target of miR-122. The restoration of miR-122 expression terminated the migration of HCC cell and the in vivo tumor expansion and prompts the apoptosis by its direct and particular control of AKT3. However, multiple targets have been investigated for miR-122 till date and in no way can completely report for the varied range of cellular modification and tumorigenic behavior, which is identified in the miR-122 downregulated HCCs.

In this research, we show the direct targeting behavior of miR-122 over AKT3 to control the cellular modifications in the tumorigenesis in the non-HCV-altered standard human HCC cell lines. Moreover, the repairing miR-122 expression in these cell lines prompts apoptosis along with hindered migration and considerably restrains the tumorigenesis. Because the phenotype prompted by the miR-122 overexpression was saved by the temporary appearance of abnormal AKT3, we present the control of AKT3 expression by miR-122 is essential and adequate for attuning tumorigenesis and the cellular modification in human HCC cell lines. The research of siRNA and gene knockout on the AKT2 and AKT1 uncovered the isoform particular roles of the AKT class members in the adjustment of cell relocation that usually associates with the capturing of tumor and the metastasis, but limited information about the role of AKT3 in the cell relocation is known. Moreover, these three isoforms of AKT are capable of transforming cells, but in vitro, expansion or gene mutation of AKT3 has still not been documented in the human cancers. There are a wide number of latest publications focusing on the role of HBV enhancing the expression of the mTOR and PI3K/AKT pathways. In our study, we demonstrate the upgraded AKT3 expressions which are responsible to control tumorigenesis in the category of highly energetic and modified HCCs. From our study, the data evidently reflects the targeting behavior and the downregulation by the miR-122 overexpression on AKT3 and can hinder relocation which is saved by the reimposition of AKT3 expression. The presence of AKT1 and AKT2 expression in the SNU-182 cells is inadequate to control the relocation and metastasis in few HCCs.

## 5. Conclusion

To conclude, we have demonstrated the direct binding by miR-122 to the 3′-UTR of the human AKT3 and the overexpression miR-122 in the HBV-altered HCC cell lines which is efficient to reduce AKT3, at transcript as well as the protein level in order to obstruct the cell relocation, prompting the apoptosis and hindering the cell growth as well as the tumor growth in the mice. The abnormally expressed AKT3 is efficient to save these antitumor behaviors prompted by the miR-122 overexpression signifying the control by miR-122 which is settled via direct targeting AKT3 in these HCC cell lines.

## Figures and Tables

**Figure 1:** Measurement of luciferase activity by SNU-182 and Huh-7.

**Figure 2:** Transcript level of AKT3 was normalized in the liver, and expression of miR-122 was measured in HCC cell lines.

**Figure 3:** Monitoring of relative expression levels in HCC cell lines of AKT1 and AKT2 (homologous isoforms).

**Figure 4:** Analysis of protein levels of AKT and AKT3 in Western blot analysis in HCC cell lines.

**Figure 5:** Western blot analysis of actin (loading control), AKT3, and total AKT protein levels in various HCC cell lines.

**Figure 6:** miR-122 overexpression and cell proliferation.

**Figure 7:** Cell migration and apoptosis in HBV-transformed HCC cell lines.

**Figure 8:** Measurement of phosphorylation of cleaved caspase 3, BAD, and total BAD in cells.

## Data Availability

The data used to support this study are available from the corresponding author upon request.
